# Oral Lichen Planus in Patients With Good’s Syndrome: A Literature Review

**DOI:** 10.7759/cureus.35177

**Published:** 2023-02-19

**Authors:** Pauline Le Gatt, Anh Tuan Nguyen, Vanessa Baaroun, Juliette Rochefort

**Affiliations:** 1 Oral Surgery, Hôpital de la Pitié-Salpêtrière/Université de Paris, Paris, FRA; 2 Dentistry, Hôpital de la Pitié-Salpêtrière/Université de Paris, Paris, FRA

**Keywords:** erosive lichen planus, oral lichen planus, lichen planus, thymoma, good syndrome

## Abstract

Good's syndrome is defined as the association of a thymoma with an immune deficiency. Many patients with Good's syndrome also have oral lichen planus involvement, and some authors have even considered it to be one of the clinical signs of Good's syndrome. In the literature, to our knowledge, clinical forms of oral lichen planus associated with Good's syndrome have not been described. We therefore aimed to characterize the forms of oral lichen planus occurring in the context of Good's syndrome. To this end, we carried out a scoping review of the literature according to the Joanna Briggs Institute guide and included 17 articles on the theme of "the forms and clinical locations of oral lichen planus associated with Good's syndrome". A total of 17 articles were selected, and 19 patients with Good's syndrome including oral lichen planus were identified. Most of them were women aged 60 years with erosive oral lichen planus of the tongue and inner cheeks. The treatments used were thymectomy, to which immunoglobulin infusions were added in some cases. All these treatments resulted in improvement of the oral lichen planus in 70.6% of cases. The management of Good's syndrome allows the improvement of oral lichen. In patients over 50 years of age with acute erosive oral lichen planus refractory to conventional therapies, Good's syndrome should be investigated.

## Introduction and background

Good's syndrome is defined as the association of a thymoma with an immune deficiency [1]. It occurs in both men and women, particularly between 40 and 50 years of age [2]. Its causes are still poorly understood, but according to some authors, the etiology of this syndrome most probably lies in the deregulation of certain cytokines that influence the growth of B and T lymphocytes [3]. Other studies consider that it is a failure of the maturation process of these same cells [4].

Many patients with Good's syndrome also have oral lichen planus involvement, and some authors have even included it as a clinical feature of Good's syndrome. This is a mucocutaneous disease with multiple clinical forms, which can occur on the skin, nails, and oral and/or genital mucosa. Localization in the oral cavity is not uncommon [5]. Several types of oral lichen planus can be distinguished: reticular, papular, plaque, erosive, atrophic, sclerotic, or bullous [5,6]. A recent classification developed by the French association named Groupe d'Etude de la MUqueuse Buccale (GEMUB) has classified oral lichen planus lesions into three categories: strict lichen planus (SLP), lichenoid lesions (LLs), and induced lichenoid lesions (ILLs) [5].

In the literature, to our knowledge, clinical forms of oral lichen planus associated with Good's syndrome have not been described. We therefore wanted to know whether these oral lichen planus lesions were SLP, LLs, or ILLs. In addition, the course of this condition after management and treatment of Good's syndrome has not been studied, and we were interested to know whether oral lesions were resolving after management and treatment of Good's syndrome.

To this end, we conducted a literature review on the subject and listed the clinical cases reported in the literature of patients with Good's syndrome including oral lichen planus involvement. The null hypothesis was that patients with Good's syndrome have an unremarkable, possibly independent oral lichen planus that does not resolve after treatment for Good's syndrome.

## Review

Materials and methods

Objectives

The primary objective of this review was to study the forms and types of oral lichen planus associated with Good's syndrome in order to determine which type of oral lichen planus was found in these clinical situations. The secondary objective was to analyze the evolution of oral lichen planus after treatment of Good's syndrome.

The main research question was: Are there any specificities regarding the clinical features (forms and locations) of oral lichen planus found in patients with Good's syndrome?

Methology of the Scoping Review

This is a scoping review of the literature according to the Joanna Briggs Institute guide [7]. The methodology of the Scoping Review met PRISMA requirements (Figure 1). We conducted an extensive literature search using the PubMed and Scopus bibliographic databases. Searches on Encyclopédie Médico-Chirurgicale (EMC), Journal of Oral Medicine and Oral Surgery (JOMOS), and Cochrane did not allow us to select additional articles.

**Figure 1:** PRISMA framework.

The most relevant search equation entered on Pubmeb was the following: "((((good's-syndrome) OR (good-syndrome)) OR (good-syndrome)) OR (thymoma)) AND (((((((((((lichen planus) OR (oral lichen planus)) OR (lichenoid)) OR (oral manifestation)) OR (erosive lesion)) OR (oral erosive lesions)) OR (mucosal manifestation)) OR (cutaneomucosal)) OR (mucosal lesion)) OR (oral cavity)) OR (mouth))"

A double search and double selection were performed by two people separately and independently. At each stage, in case of disagreement in selection, a third person determined the inclusion or not of the article concerned after discussion. After exclusion of duplicates, the titles and abstracts of articles were evaluated in accordance with the inclusion and exclusion criteria. Potentially eligible articles were then subject to evaluation of the full text.

The bibliographic sources of the selected articles were analyzed to include additional articles not identified by our equation. The search period defined was from January 01, 1960, to May 25, 2022.

 Inclusion Criteria

The following articles were included in our literature review: articles answering the research question based on the title and the abstract, articles available in full text from the subscriptions of each (university, INSERM, CNRS, hospitals, etc.), clinical trials, systematic reviews with meta-analyses, case series of more than one case, recommendations for clinical practice, consensus conferences, institutional publications, and medical decision articles, all containing an abstract.

Exclusion Criteria

The following articles were excluded from our literature review: articles written in a language other than English and French, duplicates within the same database and then adding up the searches on the different databases using bibliographic reference management software (Zotero), articles not mentioning Good's syndrome or oral lichen planus, and articles with no full text available.

Data Extraction

Data extraction is presented in Table 1, which includes authors and date of publication, patient age and gender, location and type of oral lichen planus, Good's syndrome treatment, and whether or not the lichen planus resolved after Good's syndrome treatment.

**Table 1:** Description of clinical data of patients with Good's syndrome associated with oral lichen planus. NC, not communicated; GS, Good's syndrome; IgG, immunoglobulin infusion; Surg, surgical thymectomy; CTC, corticosteroids

Authors and date	Age	Gender	Localization	Type of oral lichen planus	Good’s syndrome treatment	Resolution after Good’s syndrome treatment
Luque-Luna et al. (2021) [8]	NC	NC	NC	Erosive	Surg + IgG	No
Kaku et al. (2011) [9]	71	F	Lips, tongue, cheeks	Erosive + plaque	Surg + local CTC + retinoids	No
Blanchard et al. (2010) [2]	85	F	Tongue, cheeks	Erosive + reticulation	Surg + local CTC + IgG after improvement	Yes
Motegi et al. (2015) [10]	59	M	Lips, tongue, cheeks	Erosive	Local CTC + local tacrolimus	No
Ni et al. (2021) [11]	70	F	NC	NC	Surg	NC
Seneschal et al. (2008) [3]	68	M	Tongue, cheeks	Erosive + reticulation	Surg + oral and local CTC + oral retinoids + local tacrolimus	No
Maehara et al. (2015) [12]	48	F	Tongue, cheeks	Erosive + plaque	Surg + IgG	Yes
Maehara et al. (2015) [12]	52	F	Tongue, cheeks	Erosive	Surg + IgG + local CTC	Yes
Macdonald et al. (2014) [13]	70	F	Tongue, gingiva, cheeks	Erosive	Surg + IgG + oral CTC + cyclosporine	Yes
Moutasim et al. (2008) [14]	54	F	Tongue, gingiva	Erosive	Oral CTC + local tacrolimus	Yes
Fatrez et al. (2020) [15]	65	F	Tongue	Erosive	Surg + local CTC + oral CTC	No
Arnold et al. (2015) [16]	40	F	Cheeks	Erosive	Surg + local CTC	Yes
Arnold et al. (2015) [16]	54	M	Tongue, cheeks	Erosive	Surg + oral CTC + cyclosporine	Yes
Tan (1974) [17]	67	M	Lips, tongue, cheeks	Erosive	Surg + oral CTC	Yes (but recurrence)
Hon et al. (2006) [18]	66	F	Tongue	Erosive	Surg + oral CTC + colchicine	Yes
Furukawa et al. (2018) [4]	74	F	NC	Reticulation	Surg	NC
Pons Benavent et al. (2021) [19]	67	M	Tongue	Erosive + reticulation	Surg + local CTC + oral tacrolimus	Yes
Flamenbaum et al. (1982) [20]	53	M	NC	Erosive	Surg + local CTC + oral CTC	Yes
Agarwal et al. (2007) [21]	53	F	NC	Erosive	Surg + oral CTC + cyclosporine	Yes

Results

Description of the Selected Articles

By conducting our search on the PubMed database, we obtained 125 articles. Using the same keywords and in the same order as for PubMed, the transdisciplinary database Scopus allowed us to obtain 177 articles (Figure 1). Adding the data obtained from the four database queries, we obtained 302 articles (Figure 1).

After eliminating duplicates (n=175), and then eliminating non-French and non-English speaking articles (n=6), we proceeded to eliminate articles without an abstract or without access to the full text (n=5), or with titles that were not relevant (n=67) or abstracts that were not relevant (n=15), and unsatisfactory methodologies or analyses outside our subject (no survival study or no discussion of risk factors) (n=20); then, after adding three articles listed in the bibliographic references of the selected articles, we included 17 articles on the theme of "the clinical forms and locations of oral lichen planus associated with Good's syndrome" (Figure 1).

Clinical Aspect of Oral Lichens Reported in Patients With Good's Syndrome

From the 17 selected articles, we identified 19 patients with Good's syndrome who had oral lichen planus (Table 1).

The majority of patients (67%) were women (12 women and 6 men) with an average age of 60.6 years at the time of diagnosis of Good’s syndrome (average calculated on 18 patients, where information was available). For one of the 19 patients, no epidemiological information was provided. The most common ethnicities were Caucasian or Asian. Patients' comorbidities were not described in most cases (Figure 2).

**Figure 2:** Epidemiological aspects of patients with oral lichen planus in Good’s syndrome. (A) Gender distribution. (B) Histogram of the distribution of the number of patients per 10-year age group.

The most frequent type of lichen planus was erosive and concerned 89% of patients. The two other forms found were hyperkeratotic plaque (11%) and reticulated plaque (21%). Different clinical forms could be found in the same patient. It was not specified whether inducing factors were identifiable (Figure 3A). Most often, patients had multiple locations at different sites. In 72% of patients, the tongue was the most common site of involvement, followed by the inside of the cheeks (53%), the lips (16%), and the gums (10%). Almost half (42%) of the patients had extra oral involvement. There was no information on the location of five (26%) of the patients (Figure 3B).

**Figure 3:** Clinical aspects of oral lichen planus reported in the literature in patients with Good's syndrome. (A) Type of lesion. (B) Localizations.

Therapeutics Used and Course of Oral Involvement

Different treatments for oral lichen planus and Good's syndrome were undertaken in the patients described in the literature. The authors also assessed the therapeutic efficacy on the improvement or not of the oral lichen planus following the treatments. It appears that the best responses are obtained after treatment with IgG infusions is added to the thymectomy.

Management of Good's Syndrome

Considering the 19 patients listed, 17 patients were treated with thymectomy. Only one of the patients did not undergo this procedure. For the last patient, no information is provided. Of the 17 patients who were treated with thymectomy, three had thymectomy before the discovery of their oral lichen planus. Of the remaining 14 patients with oral lichen planus at the time of surgery, four (28.6%) patients had an improvement in their oral lichen planus and eight (57%) patients had no improvement. No information was given on the evolution of the oral lesions for two (14.3%) patients. Of the 17 patients identified who had undergone thymectomy, five also received immunoglobulin infusions. Three of the patients who received immunoglobulin injections had an improvement in their oral lichen planus (60%), and only one had no improvement (20%). The last patient received immunoglobulin infusions at a distance from the thymectomy and local treatment of the oral lichen planus, and thus no conclusion can be drawn as to the effect on the lichen planus, as improvement of the lichen planus had already been observed before.

Management of Oral Lichen Planus

In addition to the management of thymoma, oral and local corticosteroids were the most frequently used treatments for oral lichen planus (89%). Some local immunosuppressive drugs (21%) or oral drugs such as tacrolimus, colchicine, or cyclosporine (32%) were found. If we group together all the patients who did not have a thymectomy, who did not have an improvement of their oral lichen planus following thymectomy, or who had a thymectomy before the appearance of the lichen planus, we obtain a total of 12 patients. Of these, five improved with the use of these local treatments (42%) and six did not improve (50%). There is no information on any treatments or their effects in any of the patients described. In total, five out of 17 patients had no improvement in their oral lichen planus condition, regardless of the therapy used. Thus, 70.6% of the patients (n=12) showed improvement.

Oral Lichen Planus as a Diagnostic Gateway to Good's Syndrome?

The discovery of oral lichen planus most often precedes the diagnosis of Good's syndrome (74%) and constitutes a diagnostic gateway. In fact, oral lichen planus was diagnosed after Good's syndrome in three (16%) patients, and in only one patient, oral lichen was discovered after thymoma and before hypogammaglobulinemia (5%). There is no information on the diagnostic temporality of one of the patients. Oral lichen planus may therefore be the first clinical sign of Good's syndrome and is the diagnostic gateway in the majority of cases.

Discussion

This study showed that patients with oral lichen planus in Good's syndrome were predominantly women aged around 60 years. The most common type of oral lichen was erosive and usually located on the tongue and inner cheeks. The treatments used were thymectomy supplemented by immunoglobulin infusions for five patients, combined with local treatments for 15 patients (corticosteroids, tacrolimus, or others). Tacrolimus can cause renal failure, gastrointestinal, cardiac, ocular, and opportunistic infections, and thrombotic microangiopathies. Lymphoproliferative syndromes associated with Epstein-Barr virus (EBV) have been reported in some patients, and tacrolimus can cross the feto-placental barrier, posing a risk to the fetus. People prescribed tacrolimus should be monitored with caution. Together, these treatments led to an improvement of the oral lichen in 70.6% of cases. It is important to note that 66% of the patients who underwent thymectomy associated with immunoglobulin infusions had an improvement in their oral involvement without any local treatment. Two of the 17 patients had perceived improvement in oral lichen after thymectomy alone. Most (75%) patients who had thymectomy combined with immunoglobulin infusions had improvement in their oral lichen. No improvement in oral lichens was seen in patients who did not undergo thymectomy. The combination of thymectomy and corticosteroid treatment is most often correlated to improvement of oral lichen in patients with Good's syndrome. Finally, for 75% of the patients, oral lichen planus is diagnosed before Good's syndrome and constitutes a diagnostic gateway.

Few patients could be included in this study. This is mainly due to the fact that Good's syndrome is a rare condition (ORPHA:169105) and is often studied in association with paraneoplastic autoimmune syndrome (PAMS) and multivisceral autoimmune syndrome (TAMA), from which it is not distinguished in some works. In addition, we did not include patients with extraoral lichen planus, nor those with thymoma only, without hypogammaglobulinemia. Thymoma is a malignant or benign tumor of the thymic epithelial cells and can be associated with many immune disorders [22]. In Good's syndrome, it is associated with hypogammaglobulinemia as well as few or no circulating B cells and an abnormal CD4+/CD8+ T cell ratio [22]. An association has also been observed between the presence of an isolated thymoma (without Good's syndrome) associated with oral lichen planus described in 13 patients in the literature [22], i.e., in a smaller number of patients than that reported in association with Good's syndrome, even though the incidence of thymoma (0.14/100,000 in Europe) is higher than the incidence of Good's syndrome (241 cases reported in 2022) worldwide [23]. Oral lichen planus is therefore more related to the association between thymoma and hypogammaglobulinemia than to thymoma alone.

The erosive form was the most common type of oral lichen planus in our patients with Good's syndrome (17/19 or 89%). In the general population, where the prevalence of oral lichen planus is estimated to be between 0.1% and 2.2% [24], the reticular form of oral lichen planus is much more common than the erosive form. However, the latter predominates in published work, most likely due to recruitment bias, as erosive forms are much more often symptomatic and therefore managed and published [24]. Indeed, only patients diagnosed with Good's syndrome and presenting with oral pain were considered by the authors of the 17 case reports included in our scoping review. This constitutes a recruitment bias. It is possible that patients with Good's syndrome also have lichen planus reticularis without symptoms. But no study has systematically analyzed the oral mucosa of all patients with Good's syndrome.

Lichen planus is an autoimmune disorder, related to a dysregulation of lymphocytes, especially CD8+ T cells and CD4+ T cells [20]. Good's syndrome associates thymoma with hypogammaglobulinemia and an abnormal CD4+/CD8+ T cell ratio [22]. The presence of oral lichen planus could therefore be directly related to this T-cell imbalance. This is supported by the fact that thymectomy alone does not resolve the oral lesions, as only 28.6% of patients report improvement after thymectomy (n=14). However, patients who received immunoglobulin infusions reported improvements in their oral lichen planus in 75% of the cases. However, only five patients who received these treatments have been reported in the literature. In addition, little information on the immunoglobulin levels is found in patients with Good's syndrome. In a systematic review of the literature by Shi and Wang on Good's syndrome published in 2021 (not looking at the presence of oral lichen planus) and including 162 patients, the median IgG level was 322 mg/dL (interquartile range: 188-476 mg/dL). No details of IgA and IgM levels were found [25]. Of the 11 patients in our literature review for whom IgG levels were reported, the mean level was similar to and 344.6 mg/dL. Thus, it would be interesting to conduct a prospective study on these patients to assess the impact of immunoglobulin infusion associated with thymectomy and to evaluate whether or not the initial immunoglobulin levels correlate to the presence of oral lichen planus.

Finally, our review of the literature showed that the diagnosis of oral lichen planus most often precedes that of Good's syndrome (74%) and constitutes a diagnostic entry point. Most patients are women, with an average age of 60 years, presenting with oral lichen planus, mainly erosive on the back of the tongue or the inner side of the cheeks, and refractory to conventional treatments (corticosteroids).

Screening for Good's syndrome could be proposed to patients with this clinical profile. This would include a chest X-ray and a circulating immunoglobulin test. We have proposed a decision tree that can be applied in these situations (Figure 4).

**Figure 4:** Diagnostic decision tree for Good's syndrome in oral lichen planus.

This study has some biases. Indeed, the clinical and histological descriptions of the pathologies were practitioner-dependent, and only the information cited by the authors could be taken into account. However, we ensured that the samples of the included studies were independent, i.e., that there was no overlap between the clinical cases presented. As these were only clinical case reports, this analysis did not require counting or analysis of the degree of variation in the distributions. In addition, the data were not always accessible. In particular, for one patient, the authors did not report any clinical data.

## Conclusions

Our study identified 19 patients, mostly women over 50 years of age, with Good's syndrome and lesions that were mostly erosive in nature. Thymectomy alone did not resolve the lesions. It might be interesting to carry out a prospective study on a group of patients with Good's syndrome without prior inclusion bias regarding the symptomatology of oral lesions. This would allow the prevalence of oral lichen planus involvement in this condition to be assessed and all its features to be recorded. In the case of a patient over 50 years of age with acute erosive oral lichen planus refractory to conventional therapy, Good’s syndrome should be investigated.
